# The Significance of Screening for Microvascular Diseases in Chinese Community-Based Subjects with Various Metabolic Abnormalities

**DOI:** 10.1371/journal.pone.0097928

**Published:** 2014-05-16

**Authors:** Can Pang, Lili Jia, Xuhong Hou, Xin Gao, Wei Liu, Yuqian Bao, Weiping Jia

**Affiliations:** 1 Department of Endocrinology and Metabolism, Shanghai Clinical Center for Metabolic Diseases, Shanghai Key Laboratory of Diabetes Mellitus, Shanghai Diabetes Institute, Shanghai Jiaotong University Affiliated Sixth People's Hospital, Shanghai, China; 2 Department of Ophthalmology, Shanghai Jiaotong University Affiliated Sixth People's Hospital, Shanghai, China; 3 Department of Endocrinology and Metabolism, Fudan University Affiliated Zhongshan Hospital, Shanghai, China; 4 Department of Endocrinology and Metabolism, Shanghai Jiaotong University Affiliated Renji Hospital, Shanghai, China; University of Hong Kong, CHINA

## Abstract

**Background:**

To assess the association of albuminuria and retinopathy with metabolic syndrome (MetS) and the related metabolic components defined by various criteria in Chinese community-based subjects.

**Methods:**

A total of 3240 Chinese subjects were recruited from urban communities and classified into subgroups with isolated or concomitant state of the two microvascular diseases. MetS was defined according to the standard of International Diabetes Federation, the National Cholesterol Education Program's Adult Treatment Panel III and Chinese Diabetes Society (CDS), separately. Albuminuria was defined as an elevated morning urine albumin-to-creatinine ratio. Retinopathy were identified with nonmydriatic retinal photographs according to the Diabetic Retinopathy Disease Severity Scale. Logistic regression was performed to analyze the contributive risk factors.

**Results:**

The subgroup of isolated retinopathy was the oldest (P<0.05), with higher blood pressure (*P*<0.001) and larger waist circumference (*P*<0.05). After adjusting for age, sex and other metabolic components, individuals with blood pressure over 130/85 mmHg were prone to have isolated albuminuria (OR: 1.51, *P* = 0.0001); while individuals with fasting plasma glucose over 5.6 mmol/L were in high risk of retinopathy concomitant with albuminria (OR: 3.04, *P* = 0.006). Larger waist circumference was a potential risk factors for isolated albuminuria and isolated retinopathy, though not significant after further adjustment of other metabolic components. The risk for albuminuria and retinopathy increased with the aggregation of three or more metabolic components. However, the MetS per se did not have synergic effect and only the MetS defined by CDS remained as a risk factor.

**Conclusions:**

Albuminuria and retinopathy were highly associated with accumulated metabolic abnormalities including sub-clinical elevated blood pressure and elevated fasting plasma glucose.

## Introduction

The Metabolic Syndrome (MetS) is a constellation of obesity, glucose intolerance, hypertension, hyperinsulinemia and dyslipidemia, which contributes high risk for cardiovascular diseases. Besides macrovascular complications, there was growing evidences that metabolic syndrome (MetS) is also a strong independent indicator of microvascular complications in Caucasians [1]–[6]. However, the relationship between MetS and microvascular diseases remains controversial in Asian population. In Israel, MetS using the definition of National Cholesterol Education Program's Adult Treatment Panel III (ATP III) was associated with a significantly higher risk of retinopathy and nephropathy [7]. In India, although the presence of MetS defined by International Diabetes Federation (IDF) was not significantly associated with microvascular complications in subjects with type 2 diabetes, the clustering of MetS components led to an increase in the prevalence of diabetic nephropathy[8]. Iwasaki et al found that neither the IDF definition nor the ATP III criteria of MetS increased the risk of microvascular complications in Japanese patients with type 2 diabetes[9]. However, another population based study in Japan observed that MetS defined by IDF was associated with microvascular changes in the retina [10]. Such discrepancies were considered partly to be attributed to the ethnic variances.

The worldwide concepts of MetS according to the currently available criteria were originated mostly from European- or American-based data[11], [12]. It still remains questionable as to whether they are applicable to evaluate the risk of diabetic microvascular complications in Chinese population. Hence, in the present study, we aimed to assess the association of albuminuria and retinopathy with MetS in Chinese community-based subjects and evaluate the contributive efficacy of various MetS defined criteria and the related metabolic components to the diabetic microvascular diseases.

## Materials and Methods

### Study population

All the protocols associated with this study were approved by the Human Research Ethics Committee of Shanghai Sixth People's Hospital and all the reported investigations have been carried out in accordance with the principles of the Declaration of Helsinki as revised in 2000. Written informed consent was obtained from each patient in duplicate and separately held by the patient and investigators. The consent procedure was approved by the above ethics committee. Shanghai Diabetic Complications Study (SHDCS) was communty-based study to screen for microvascular and macrovascular complications in Chinese aged over 20 years. The study population and methods have been described in detail previously [13], [14]. A total of 3714 residents in four adjacent located communities (Caoyang, Huayang, Changfeng, Tangqiao) were recruited between 2005 and 2007. Subjects with type 1 diabetes, acute renal failure or those receiving dialysis were excluded. Informed consent was obtained from all participants. Each participant received a 75 g oral glucose tolerance test, except for those with a validated history of diabetes mellitus. Of these 3714 subjects, those without retinal examintation (n = 217) or urine test (n = 19), or with retinal photographs of insufficient quality for grading (n = 238) were excluded, leaving 3240 identified as eligible.

### Anthropometric measurements and biochemical assay

Blood pressure (BP) was taken three times using a standard mercury sphygmomanometer and then averaged. Body mass index (BMI) was calculated as weight divided by height squared (kg/m^2^). The waist-to-hip ratio was calculated as the ratio of the waist circumference to the hip circumference.

Plasma glucose levels were measured using the glucose oxidase method. Glycated haemoglobin (HbA_1c_) was measured by high performance liquid chromatography (HLC-73G7, Tosoh, Japan) [15]. The Shanghai Diabetes Institute successfully participated in the HbA_1c_ Quality Assessment Program of the Chinese Ministry of Health between 2006 and 2008. The HbA_1c_ inter-assay and intra-assay coefficients of variation were <0.4%, and <0.6%. Lipid profiles, including total cholesterol, triacylglycerol, high density lipoprotein [HDL]-cholesterol and low density lipoprotein [LDL]-cholesterol, were measured on a Hitachi 7600 analyser using an enzymatic assay. Hypersensitive C-reactive protein (CRP) was examined by nephelometry (Vista CardioPhase high sensitivity CRP, Dade Behring). First morning urine was collected once a month for 3 months. Urinary albumin was determined on a DADE BEHRING BN II analyser by nephelometry (N antiserum to Human Albumin Assay, Dade Behring). Urinary creatinine concentration was measured on a Hitachi 7600 analyser using the sarcosine oxidase-PAP method. All control values were consistent with the standard recommended by the Shanghai Clinical Testing Center.

### Definitions of Metabolic syndrome

Hypertension was diagnosed as systolic BP ≥140 mmHg and/or diastolic BP ≥90 mmHg. Obesity was defined as a BMI ≥30 kg/m^2^. Diabetes and IGR were diagnosed according to the standard set by American Diabetes Association. CVD was defined as coronary heart disease or stroke.

The IDF definition of MetS is central obesity (waist circumference ≥90 cm in male, ≥80 cm in female) and any two of the following[12]: (1) Triglycerides ≥1.7 mmol/L, or specific treatment for this lipid abnormality; (2) HDL cholesterol <1.03 mmol/L in male, <1.29 mmol/L in female, or specific treatment for this lipid abnormality; (3) Systolic BP ≥130 mmHg or diastolic BP ≥85 mmHg, or treatment of previously diagnosed hypertension; (4) Fasting plasma glucose (FPG) ≥5.6 mmol/L, or previously diagnosed type 2 diabetes.

The US ATP III requires at least three of the following to define MetS[11]: (1)Central obesity; (2) Triglycerides ≥1.7 mmol/L, or treatment for this lipid abnormality; (3) HDL-cholesterol <1.03 mmol/L in male, <1.29 mmol/L in female, or treatment for this lipid abnormality; (4) Systolic BP ≥130 mmHg or diastolic BP ≥85 mmHg, or treatment of previously diagnosed hypertension; (5) FPG ≥5.6 mmol/L.

The Chinese Diabetes Society (CDS) criteria for metabolic syndrome requires 3 items or all the four items[16]: (1) BMI ≥25 kg/m^2^; (2) FPG ≥6.1 mmol/L, or 2 h postprandial plasma glucose(2 hPG) ≥7.8 mmol/L, or diagnosed diabetes; (3) Systolic BP ≥140 mmHg or diastolic BP ≥90 mmHg, or treatment of previously diagnosed hypertension; (4) Triglycerides ≥1.7 mmol/L and/or HDL-cholesterol <0.9 mmol/L in male or <1.0 mmol/Lin female, or treatment for this lipid abnormality.

### Assessment of albuminuria and retinopathy

Albuminuria was defined as urine albumin-to-creatinine ratio ≥30 mg/g. Fundus photography was performed at each site following a standardized protocol. Participants were seated in a darkened room, and the posterior pole of each eye was photographed with a 45° 6.3-megapixel digital non-mydriatic camera (Canon CR6-45NM, Lake Success, New York, USA). Two independent trained readers without knowledge of the clinical details read the photographs. DR was graded according to the Diabetic Retinopathy Disease Severity Scale [17]. Grade 0: no abnormalities; Grade 1: mild non-proliferative retinopathy (microaneurysms only); Grade 2: moderate non-proliferative retinopathy (more than just microaneurysms, but less than Grade 3); Grade 3: severe non-proliferative retinopathy; Grade 4: proliferative retinopathy. Patients with both albuminuria and retinopathy were defined as concomitance of albuminuria and retinopathy.

### Statistical analysis

All analyses were performed using SPSS software version 15.0. Normally distributed and continuous variables were expressed as mean ± standard deviation, and non-normally distributed variables were presented as medians (quartiles 25% and 75%). An one-way ANOVA with SNK analysis was used to compare differences with regard to quantitative data. A Kruskal-Wallis H test was used for comparisons of non-normally distributed data. Multinominal logistic regression were performed to determine the risk factors for microvascular diseases subgroups. *P*<0.05 was considered significant (two tailed).

## Results

### Basic features

A total of 3240 participants with an average age of 60.7±11.0 years were analyzed, including 1229 males and 2011 females. Almost 20.2% of the subjects had albuminuria (n = 654) and 4.0% had retinopathy (n = 130). There were 53.2% of participants with hypertension (n = 1725), 24.5% with diabetes (n = 793), 26.6% with impaired glucose regulation (n = 863), 4.9% with obesity (n = 160), 14.4% with cardiovascular diseases (n = 458), 53.1% with dyslipidemia defined as high triglycerides, or low HDL-cholesterol, or high LDL-cholesterol in ATP III definition (n = 1691/3182).

We classified the participants into four subgroups: without albuminuria or retinopathy, isolated albuminuria, isolated retinopathy, and concomitance of albuminuria with retinopathy (Table 1). Individuals with isolated retinopathy had oldest age (*P*<0.05), highest blood pressure (*P*<0.001), larger waist circumference (*P*<0.05). The level of FPG (*P*<0.05), 2hPG (*P*<0.05), HbA_1c_ (*P*<0.05) and C-reactive protein (*P*<0.05) was highest in those with concomitance of albuminuria and retinopathy, a subgroups with highest frequency of diabetes and metabolic syndrome. Individuals with both retinopathy and albuminuria had the highest rate of known diabetes (54.5%), however in subjects with isolated retinopathy, the rate of newly-diagnosed diabetes was the highest of all. The positive rates of urine white blood cell test were similarly high between subjects without albuminuria or retinopathy (17.4%) and with isolated retinopathy (19.4%).

**Table 1:** Demographics of subjects with or without albuminuria and diabetic retiopathy.

	Absence of albuminuria or retinopathy (n = 2500)	Isolated albuminuria (n = 610)	Isolated retinopathy (n = 86)	Concomitance of albuminuria and wih retinopathy (n = 44)
**Age (years)**	60.2±11	62.4±11.2	64.5±9.8*	63.2±9.7
**Male**	1016(40.6)	160(26.2)	40(46.5)	13(29.5)
**Systolic BP (mmHg)**	129.4±18.2	134±19.1	138.7±20.5**	134.0±16.4
**Diastolic BP (mmHg)**	80.8±9.8	82.9±9.9	84.1±10.2*	81.4±9.7
**BMI (kg/m2)**	24.4±3.3	24.7±3.3	25.1±3.7	24.9±2.9
**Waist circumference (cm)**	82.1±9.5	83.3±9.4	85.6±10.7*	84.0±9.3
**WHR**	0.87±0.07	0.87±0.06	0.89±0.06*	0.88±0.06
**FPG (mmol/L)**	5.96±1.52	6.06±1.78	7.42±2.88*	8.79±3.91*
**2hPG (mmol/L)**	7.58±3.4.0	7.66±3.48	9.41±5.23*	10.54±7.78*
**HbA1_c_ (%)**	5.7(5.4–6.1)	5.8(5.4–6.2)	6.5(5.8–7.7)*	7.4(6.0–10.3)*
**Total cholesterol(mmol/L)**	4.85±1.02	5.03±1.05	4.71±0.82	5.04±0.89
**Triglyceride (mmol/L)**	1.34(0.97–1.91)	1.40(1.00–2.04)	1.31(1.04–1.86)	1.38(0.97–2.15)
**HDL-cholesterol (mmol/L)**	1.33±0.37	1.33±0.37	1.25±0.33	1.31±0.40
**LDL-c (mmol/L)**	2.92±0.97	3.02±0.88	2.83±0.67	3.06±0.80
**CRP**	0.89(0.43–1.86)	1.43(0.73–3.21)*	0.67(0.40–2.01)	2.32(0.70–4.37)*
**CVD**	321(12.8)	112(18.4)	14(16.3)	11(25)
**Current smoker**	427(17.3)	63(10.3)	7(8.1)	7(15.9)
**Hypertension**	1260(50.4)	373(61.1)	64(74.4)	28(63.6)
**Obesity**	115(4.6)	35(5.7)	9(10.5)	1(2.3)
**Diabetes**	558(22.3)	161(26.4)	46(53.5)	28(63.6)
** Known**	295(11.8)	93(15.2)	33(38.4)	24(54.5)
** Newly-diagnosed**	263(10.5)	68(11.1)	13(15.1)	4(9.0)
**IGR**	696(27.8)	145(23.8)	17(19.8)	5(11.4)
**Urine test**	1439(57.6)	217(35.6)	58(67.4)	27(61.4)
** WBC positive**	251(17.4)	42(19.4)	8(13.8)	3(11.1)
**Metabolic syndrome**				
** IDF**	781(31.5)	230(38.4)	38(44.2)	21(48.8)
** ATP III**	1069(43.3)	298(50.4)	49(57)	26(61.9)
** CDS**	761(30.6)	223(37.0)	41(47.7)	21(48.8)

Categorical variables were expressed as numbers (percentage).

Continuous variables were expressed as mean ± standard deviation or median (25% and 75%quartile) for non-normally distributed variables.

BMI, body mass index; BP, blood pressure; CVD,cardiovascular disease; FPG, fasting plasma glucose; 2hPG, 2-hour postprandial plasma glucose; HbA1_c_, glycated hemoglobin A1c; HDL, high density lipoprotein; LDL, low density lipoprotein.

*P<0.05,

**P<0.01 comparison with subgroup of absence of albuminuria or retinopathy using an one-way ANOVA with SNK analysis in regard to quantitative data and a Kruskal-Wallis H for non-normally distributed data.

According to the various criteria, the frequency rate of MetS was 33.3% by IDF, 45.2% by ATP III and 32.5% by CDS. There were no significant difference in the prevalence rate of albuminuria and retinopathy among subjects with the various MetS definitions, as shown in Table 2.

**Table 2:** Frequency of albuminuria and/or retinopathy in subjects with or without various definitions of metabolic syndrome.

	Definitions	N	Isolated albuminuria	Isolated retinopathy	Concomitance of albuminuria wih retinopathy
With MetS	IDF	1070	230(21.5)	38(3.6)	21(2.0)
	ATP III	1442	298(20.7)	49(3.4)	26(1.8)
	CDS	1046	223(21.3)	41(3.9)	21(2.0)
P value			0.863	0.785	0.925
Without MetS	IDF	2140	369(17.2)	48(2.2)	22(1.0)
	ATP III	1745	293(16.8)	37(2.1)	16(0.9)
	CDS	2175	380(17.5)	45(2.1)	22(1.0)
P value			0.852	0.922	0.934

MetS, metabolic syndrome.

In 445 subjects with known diabetes, those using anti-diabetic drugs (n = 309) had significantly higher level of FPG (8.7±2.6 vs. 7.5±2.4 mmol/L, P<0.0001), 2hPG (15.2±5.5 vs. 13.6±5.2 mmol/L, P = 0.129) and HbA_1c_ (7.6±1.7 vs. 6.8±1.5%, P<0.0001) than those without drug treatment. In 880 patients with known hypertension, those using anti-hypersensitive drugs had significantly higher systolic BP (143.8±17.4 vs. 139.9±17 mmHg, P = 0.024), but the same level of diastolic BP (87.3±10.1 vs. 87.3±9.4 mmHg, P = 0.988) compared with those without treatment. In 535 subjects with known dyslipidemia, those using lipid lowering drugs had significantly higher triglycerides (2.86±1.85 vs. 2.28±1.43 mmol/L, P = 0.047) and lower HDL-cholesterol (1.07±0.23 vs. 1.24±0.37 mmol/L, P<0.0001) than those without drug treatment.

### The association of albuminuria and retinopathy with metabolic syndrome and its components

After adjusting for age and sex (Table 3, model 1), individuals with larger waist circumference or higher blood pressure (over 130/85 mmHg) in IDF/ATPIII definition were more likely to have isolated albuminura or isolated retinopathy. The elevated fasting plasma glucose (over 5.6 mmol/L) positively correlated with high risk of retinopathy with (OR: 1.71, *P* = 0.027) or without albuminuria (OR: 3.12, *P* = 0.003). After further adjusting for other components of the metabolic syndrome (Table 2, model 2), only two associations remained significant: higher blood pressure with isolated albuminuria (OR: 1.51, *P*<0.0002), elevated FPG with the coexistence of albuminuria and retinopathy (OR: 3.04, *P* = 0.006).

**Table 3:** The association of metabolic syndrome with albuminuria and retinopathy.

	Isolated albuminuria		Isolated retinopathy		Albuminuria combined with retinopathy	
	Adjusted odds ratio (95%CI)		Adjusted odds ratio (95%CI)		Adjusted odds ratio (95%CI)	
	Model 1	Model 2	Model 1	Model 2	Model 1	Model 2
**MetS (IDF)**	1.15(0.95–1.39)		1.60(1.02–2.5)*		1.79(0.96–3.34)	
**MetS (ATP III)**	1.16(0.96–1.40)		1.53(0.98–2.38)		1.85(0.97–3.53)	
**Waist circumference ≥90 cm (male), ≥80 cm (female)**	1.24(1.04–1.50)*	1.13(0.93–1.38)	1.59(1.02–2.48)*	1.52(0.95–2.41)	1.54(0.82–2.86)	1.36(0.70–2.66)
**Triglyceride ≥1.7 mmol/L**	1.13(0.93–1.36)	1.03(0.84–1.26)	0.74(0.47–1.19)	0.57(0.35–0.94)*	0.81(0.42–1.57)	0.58(0.29–1.17)
**HDL-cholesterol <1.03 mmol/L (male), <1.29 mmol/L (female)**	1.13(0.94–1.36)	1.10(0.90–1.34)	1.20(0.77–1.87)	1.21(0.76–1.93)	1.29(0.69–2.41)	1.24(0.64–2.39)
**Blood pressure≥130/85 mmHg**	1.49(1.22–1.82)**	1.51(1.22–1.86)*	1.79(1.07–3.01)*	1.68(0.99–2.86)	1.75(0.87–3.52)	1.79(0.83–3.84)
**FPG≥5.6 mmol/L**	0.90(0.75–1.08)	0.84(0.69–1.02)	1.71(1.06–2.74)*	1.60(0.99–2.58)	3.12(1.48–6.59)**	3.04(1.37–6.74)**
**MetS (CDS)**	1.24(1.03–1.51)*		1.80(1.16–2.79)**		2.02(1.09–3.77)*	
**BMI≥25.0 kg/m2**	1.11(0.93–1.33)	1.02(0.84–1.24)	1.12(0.73–1.73)	0.93(0.59–1.46)	1.68(0.92–3.06)	1.51(0.79–2.89)
**Blood pressure≥140/90 mmHg**	1.57(1.30–1.90)**	1.59(1.30–1.95)**	2.31(1.42–3.77)**	2.25(1.36–3.73)**	1.61(0.85–3.05)	1.45(0.73–2.89)
**Triglyceride ≥1.7 mmol/l, or HDL-cholesterol<0.9 mmol/L(male), <1.0 mmol/L(female)**	1.18(0.98–1.42)	1.12(0.92–1.36)	0.90(0.58–1.41)	0.70(0.44–1.11)	1.00(0.53–1.89)	0.71(0.36–1.37)
**IGR or diabetes**	0.94(0.78–1.13)	0.85(0.69–1.03)	2.33(1.42–3.84)**	2.22(1.33–3.7)**	2.88(1.42–5.83)**	3.17(1.45–6.93)**

Model 1, adjusted for age and sex. Model 2, adjusted for age, sex, and all other metabolic components. CI, confidence interval. IGR, impaired glucose regulation.

*P<0.05,

**P<0.01.BMI, body mass index; CI, confidence interval; FPG, fasting plasma glucose;HDL, high density lipoprotein; IGR, impaired glucose regulation; MetS, metabolic syndrome.

The MetS definition of CDS per se significantly indicated higher risk for albuminura and/or retinopathy. After adjusting for other metabolic components, blood pressure over 140/90 mmHg (OR: 2.25, *P* = 0.002) and the presence of IGR or diabetes (OR: 2.22, *P* = 0.002) were the two remained independently risk factors for isolated retinopathy. Patients with hypertension (over 140/90 mmHg) were prone to have isolated albuminuria (OR: 1.59, *P*<0.0001), and hyperglycemia (IGR or diabetes) was signifianctly associated with the coexistence of albuminuria and retinopathy (OR: 3.17, *P* = 0.004).

### Increased risk of albuminuria and retinopathy with cumulative metabolic components

The risk for albuminuria and retinopathy in those with MetS was significantly elevated with the increment of metabolic components (Table 4). The aggregation of 5 metabolic components in IDF/ATPIII definition increased 1.6 times and 3.4 times risk for albuminurai and retinopathy than those without MetS. As high triglyceride (>170 mg/dl) was a negative contributive factor for retinopathy and separated from low HDL-cholesterol as an independent metabolic components in IDF/ATPIII definition, the cumulative risk of metabolic components in IDF/ATPIII definitions was not in the same order of magnitude as that in CDS definition, in which high triglyceride and low HDL-cholesterol were united into one components.

**Table 4:** Contribution of cumulative metabolic components in albuminuria and retinopathy.

Number of metabolic component		Isolated albuminuria			Isolated retinopathy		
		N	Odds ratio (95%CI)	*P*	N	Odds ratio (95%CI)	*P*
IDF/ATPIII	5	65	2.6(1.7–3.9)	0.000	13	4.4(1.6–11.9)	0.003
	4	99	1.5(1.1–2.2)	0.021	8	1.1(0.4–3.1)	0.889
	3	131	1.4(1.0–2.1)	0.038	28	2.7(1.1–6.6)	0.030
	2	144	1.4(1.0–1.9)	0.069	21	1.7(0.7–4.4)	0.236
	1	97	1.2(0.8–1.7)	0.342	10	1.1(0.4–3.0)	0.901
	0	5	1		6	1	
CDS	4	86	1.8(1.3–2.5)	0.000	13	3.3(1.4–8.1)	0.009
	3	134	1.3(1.0–1.7)	0.097	28	3.2(1.5–7.2)	0.004
	2	144	1.2(0.9–1.5)	0.295	21	2.1(0.9–4.7)	0.086
	1	127	1.0(0.8–1.4)	0.930	16	1.5(0.7–3.6)	0.318
	0	97	1		8	1	

CI, confidence interval.

## Discussion

The present study showed that metabolic syndrome defined by Chinese Diabetes Society was highly associated with albuminuria and retinopathy in Chinese subjects rather than IDF or ATP III definition. We confirmed that hypertension and hyperglycemia were the two contributive factors for isolated albuminia and retinopathy, respectively. The associations between the clustering of metabolic components with renal and retinal microvascular disease in the present study are consistent with previous studies [4], [7], [8], [18].

In our previous study regarding the risk of microvascular diseases in subjects with diabetes and impaired glucose regulation, we found that elevated blood pressure was highly associated with the presence of retinopathy in subjects with impaired glucose regulation[14]. Hypertension also indicated high risk of albuminuria in non-diabetic subjects, though not significantly[13]. As there might exist certain interference between the two microvascular diseases, we classified the participants into subgroups with isolated or concomitant state of the two microvascular diseases in the present study. An elevated blood pressure over 130/85 mmHg already indicated the high risk of albuminuria, and an individual with hypertension should be confirmed by screening as whether to have retinopathy even with diabetes or not. Only the presence of hyperglycemia suggested the concomitance of albuminuria with retinopathy.

Waist circumference was suggested to be associated with albumiunria in subjects with type 2 diabetes in Japan [18] and China [19]. The Funagata Study also confirmed positive associations between larger waist circumference defined by IDF with retinopathy after adjusting for other componentsin community-based population [10]. Our previous epidemiologic survey revealed that the peak frequency distribution of waist circumference was increased with aging [20]. The difference of waist circumference was 5 cm larger in men than in women in the age group of 50–59 years, and getting closer after 60 years. Measurement of visceral fat area using magnetic resonance imaging further suggested that the appropriate cut-offs of waist circumference might be 85 cm for the high risk of MetS in Chinese women [21]. Considering that the mean age of the participants exceeded 60 years, a modified cut-offs of waist circumference (≥90 cm in men, ≥85 cm in women) would independently increase the risk for isolated retinopathy (1.73[1.10–2.73], *P* = 0.018), even after adjusting for sex, age and other metabolic components.

Several population-based studies from the United States [22], Japan [23], Singapore [24] and rural area of China [25] have shown that CRP was associated with microalbuminuria, as is the same in our study for CRP also presented high in subjects with albuminumia. Both of albuminuria and high CRP are considered as strong and independent risk factors for CVD in patients with hypertension and diabetes as well as in the general population. A recent study even added to the fact that elevated urine albumin and high CRP could increase value to MetS variables in predicting CVD and chronic kidney disease. Different from that, isolated retinopathy were more likely to have lower level of CRP, which was consistent with the data from the Singapore Malay Eye Study [26]. In Danish type 1 diabetes, higher level of CRP was evidenced to be associated proliferative diabetes retinopathy, but this was no longer statistically significant after adjustment for diabetes duration and glycemic level [27].

The patients with albuminuria or retinopathy had higher frequency of MetS, especially in those with the concomitance. Although an increase in number of metabolic syndrome components was associated with higher likelihood of having retinopathy or albuminuria, there was no synergistic effects of MetS per se beyond individual effects of each metabolic component. The magnitude of the associations between hypertension or hyperglycemia with albuminuria or retinopathy were much stronger. Furthermore, only the metabolic syndrome per se in CDS definition was associated with both albuminuria and retinopathy. One possible explanation was the different cut-offs for elevated blood pressure and blood glucose between IDF/ATP III and CDS criteria. Furthermore, the diagnosis of MetS based on the IDF or ATP III definition was highly dependent on the waist circumference.

There were several limitations of our study should be considered. A major limitation was the use of screening methods which mignt restrict the detection rate of patients. Another limitation is the cross-sectional design of our study, in which metabolic syndrome and its components just indicated, but not predicted microvascular complications. Furthermore, a selection bias was inevitable in our study as it was not population-based and over ten percent of the recruited individuals had no retinal photographs or with ungradable photos.

## Conclusions

Microvascular diseases were prone to be present in individuals with metabolic disorders even without glycemic disorders. The risk of albuminuria and retinopathy increased with the numbers of metabolic components rather than metabolic syndrome per se. Hypertension and hyperglycemia were the two respectively independent indicators for albuminuria and retinopathy, even under subclinical abnormalities, including elevated blood pressure (over 130/85 mmHg) and elevated fasting plasma glucose (over 5.6 mmol/L). Metabolic syndrome and its components defined by CDS raised high risk for microvascular diseases in Chinese and suggested screening initiation.
